# Mechanism of miR-760 Reversing Lung Cancer Immune Escape by Downregulating IDO1 and Eliminating Regulatory T Cells Based on Mathematical Biology

**DOI:** 10.1155/2022/2960773

**Published:** 2022-07-14

**Authors:** Hong Ge, Lili Wang, Wenqiang Chen, Lei Wang

**Affiliations:** ^1^Pulmonary and Critical Care Medicine, Zibo Central Hospital of Shandong Province, Zibo, 255000 Shandong, China; ^2^Pneumology Department, Chengwu Hospital, Chengwu, China; ^3^Laboratory Medicine, Zibo Zhoucun People's Hospital, Zibo, 255300 Shandong, China; ^4^Department of Oncology, Chengyang District People's Hospital, Qingdao, 266100 Shandong, China

## Abstract

In cancer biology, mathematical models have become indispensable. They are useful for gaining a mechanistic grasp of cancer's dynamic processes. In cancer research, mathematical modelling approaches are becoming more common. The complexity of cancer is well suited to quantitative approaches as it provides challenges and opportunities for new developments (Altrock et al., 2015). *Background*. MicroRNA-760 (miR-760), as an early discovered tumor suppressor gene, is poorly expressed in lung cancer (LC). Indoleamine 2,3-dioxygenase 1 (IDO1), as an important regulator of T cell function, is active in immune tolerance. We discovered that miR-760 has a targeted relationship with IDO1, but the regulatory mechanism between miR-760 and IDO1 is still unclear. *Method*. The miR-760 and IDO1 levels in NSCLC were tested via real-time quantitative polymerase chain reaction (qRT-PCR) and western blotting (WB). Cell growth was tested by CCK8, and NSCLC cell migration and invasion were analyzed through Transwell analysis. The binding conditions and target gene of miR-451 in NSCLC cells were determined via double luciferase reporter gene. The CD8+ T and CD4+ T cell ratio in CD45+cells was assessed by flow cytometry. *Results*. qRT-PCR revealed that miR-760 was low-expressed and IDO2 was highly expressed in LC. miR-760 mimics suppressed cell growth, invasiveness, and migration. We also observed that miR-760 could downregulate the IDO1 protein level. Significantly, we revealed that miR-760 could inhibit CD8+ T cell apoptosis by controlling IDO1 enzyme function. *Conclusion*. Our findings show that miR-760 inhibits CD8+ T cell responses in LC through regulating IDO1, laying the groundwork for the development of novel vaccination therapies for the treatment of LC.

## 1. Introduction

Lung carcinoma (LC) is the most common type of cancer in people worldwide [1]. According to statistics [2], around one million new patients are admitted each year. Small cell lung carcinoma (SCLC) and non-small-cell lung carcinoma (NSCLC) are the two types of LC, with the latter accounting for approximately 85% of cases. Despite the development of numerous therapeutic options, the long-term viability of LC patients is still quite low. The prognosis of advanced or metastatic LC patients is rather poor [3]. Therefore, it is very crucial to understand the pathogenesis of LC for developing new therapeutic targets.

MicroRNA (miR) is an endogenous small noncoding RNA, 20-25 nucleotides long [4–6]. miR can control cell viability, growth, differentiation, migration, invasiveness, and metastasis through the binding of 3′-untranslated regions (UTR) of some targeted genes [7–9]. Currently, studies have shown that [10] more than 30% of human genes can be controlled by miR. Moreover, more and more studies have confirmed that [11, 12] miR affects the development and progress of various tumors through downstream target genes. miR-760 is located on human chr1 chromosome. miR-760 directly affects human carcinoma processes (such as tumorigenesis, migrations, and metastases) and regulates various tumor progression [13–15]. miR-760's mechanism in LC is still vague.

Indoleamine 2,3-dioxygenase 1 (IDO1) is a rate-limiting enzyme in tryptophan catabolism and suppresses T-lymphocytes and other immune cells [16]. Evidence showed that IDO-1 not only participates in the immune escape process of lung cancer but also contributes to the safety of the pretumor area [17]. In addition, studies have shown [18] that IDO-1 can induce immunosuppression and promote tumor progression in LC animal models. We first predicted miR-760's potential targeted genes online and concluded that miR-760 and IDO1 had a targeted binding connection. This suggested that miR-760 might affect the immune regulation of LC by targeting IDO1. Therefore, this research seeks miR-760's potential mechanism in LC, providing a new direction for clinical targeted therapy and drug development.

The arrangements of this paper are as follows: Section 2 discusses the materials and methods.  Section 3 examines a result and experiments.  Section 4 analyzes a discussion.  Section 5 concludes the article.

## 2. Methods and Materials

### 2.1. Clinical Data

From January 2014 to January 2016, fifty-two NSCLC cases in our hospital were selected, and their tumor and surrounding tissues were collected. The tissues were transited in liquefied nitrogen and conserved at -80°C for later use and unified testing. In this research, all participants had not received antitumor treatment before. Informed consent forms were obtained, and the research was ratified by the Medical Ethics Committee. This study was based on Declaration of Helsinki [19].

### 2.2. Cell Culture

Human LC cells (A549, H1975, and H1299) and bronchus epithelial cell strain HBE were from American Type Culture Collection (ATCC, Shanghai, China). The purchased cell strains were cultivated in RPMI 1640 medium comprising 10% FBS, 100 IU/ml penicillin and 100 *μ*g/ml streptomycin at 5% CO_2_ and 37°C (Invitrogen, Carlsbad, CA, the United States).

### 2.3. Cell Transfection [20]

The miR-760 mimics (miR-760-mimics), miR-760 inhibitor (miR-760-inhibit), and nonspecific control miRNA (mimics-NC/inhibit-NC) were provided by Riobio (Guangzhou, China). IDO2 sequence length was selected and pcDNA-3.1 was used as the vector. Overexpression vector of IDO2 (pcDNA-IDO2) was constructed and blank vector was used as control (pcDNA-NC) for transient transfection. Lipofectamine 2000 (Invitrogen, Carlsbad, CA) was used to inoculate cells onto six-hole culture plates. The precursor sequences of miR-760 and miR-NC (negative control) were introduced into the pLV-THM lentivirus vector to create a nude mouse tumor allogeneic model. Cotransfection of HeK-293T cells with pSPAX2, pMD2.G, and LipoFilter reagent resulted in the packaging of the recombinant lentivirus. The supernatant liquid with lentivirus particles was obtained after transfection for 48 h and 72 h and filtered and centrifuged at high speed to concentrate the recombinant lentivirus. In the presence of 5 *μ*g/ml polypropylene, lentivirus with MOI of about 5 was transduced into A549 cells. The supernatant was removed and replaced by fresh complete medium 24 h later. The infection efficiency was verified through RT-PCR after infection for 96 h. Cells were chosen with 2 *μ*g/ml puromycin for two weeks.

### 2.4. qRT-PCR [21]

The general RNA was obtained from collected tissues and cells with TRIzol (Invitrogen, the United States) agent. General RNA of each specimen was transcribed into first strand cDNA via PrimeScript™ RT Master Mix kit (TaKaRa, Tokyo, Japan). The SYBR Premix Ex Taq™ and ABI Prism 7500 detecting systems were conducted to real-time PCR, and the reaction system and reaction conditions were configured in accordance with the manufacturer's specifications. 2^-*ΔΔ*Ct^ was applied to analyze data and data processing [19]. The following are the primers: miR-760 upstream primer 5′-CGAGCGGCTCTGGGTCTG-3′and downstream primer 5′-CAGTGCAGGGTCCGAGGT-3′, U6 upstream primer 5′-GCGTCGTGAAGCGTTC-3′and downstream primer 5′-GTGCAGGGTCCGAGGT-3′, and IDO1 upstream primer 5′-AGGATGCGTGACTTTGTG-3′and downstream primer 5′-GATCTACTATTGCGAGGTG-3′. GAPDH was the inner reference of mRNA and U6 was for miR.

### 2.5. WB Experiment

The logarithmic growth phase cells were collected, and the cell concentration was adjusted to 5 × 10^5^/ml and inoculated in a 6-hole plate overnight in a 37°C, 5% CO_2_ incubator; then, the culture solution was discarded and dihydrotanshinone I solution was added dropwise with different concentrations; 100 *μ*l of culture medium was set as a blank control group and cultivated at 37°C, 5% CO_2_. It was rinsed 3 times in PBS solution, and cells were put in an EP tube, and RIPA lysate was added dropwise, 30 min later centrifuged for 15 min at 12000 r/min. The supernatant was obtained and transferred to a new EP tube. The OD value was tested via a microplate reader at a wavelength of 490 nm for protein quantitative analysis. The wet transfer method was used to transfer the protein to the nitrocellulose membrane, and 5% skim milk was added dropwise and blocked for 60 min; GAPDH was the internal reference protein, and the primary antibody was added dropwise, with a dilution ratio of 1 : 1000, and cultivated at 4°C. Subsequently, it was cleaned by PBS solution 3 times, and the corresponding secondary antibody was added dropwise, with a dilution ratio of 1 : 5000, and then sealed for 1 h. It was performed in accordance with the instructions of the ECL chemiluminescence detection kit, and a gel imaging analysis system was used to analyze the bands and determine the OD value of each band.

### 2.6. Detection of Cell Proliferating

Cell growth was tested via cell counting kit 8 (CCK-8). The brief description was as follows: the transfected cells were inoculated in 96-hole plate at 4∗10^3^ cells per hole and cultivated for 24 h, 48 h, 72 h, or 96 h. CCK-8 solution (Keygen Biotech, Nanjing, China) was put in. Then, cells were cultivated at 37°C for 60 min. The absorbance was tested at 450 nm via a spectrophotometer. Data represented three independent tests conducted in triplicate.

### 2.7. Transwell Experiment

Transwell test was employed to test cell invasiveness and migration. Matrigel (BD Biosciences, USA) was precoated in Transwell's upper chamber during invasion, but not in the upper chamber during migration. The exact procedure was as follows: the transfected cells were suspended in single cell suspension in serum-free culture media at a density of 5∗104 cells/ml in the upper chamber. A total of medium (500 *μ*l) comprising 10% FBS was put in the lower chamber. All Transwell chambers were placed 25 h at 37°C and 5% CO_2_. Invasive cells were immobilized with 4% formaldehyde and dyed with 0.1% crystal violet. Invading cells were counted under an optical microscope (Nikon, Tokyo, Japan).

### 2.8. Immunofluorescence Staining [22]

The tissue slices of nude mice with LC were obtained, dried at 60°C for 1 h, dewaxed with xylene, and rehydrated with ethanol fractionation. The antigen repair was processed with citrate buffer (pH 6.0), autoclaved and sterilized at 121°C, cleaned by PBS, and sealed 30 min with goat serum at room temperature. Then, the rat anti-mouse IDO1 and rabbit anti-mouse CD8+ antibodies were added, respectively, and kept at 4°C for one night. The slides were rinsed with PBS, and the goat anti-rabbit and anti-rat IgG second antibodies were added, respectively, and placed at ambient temperature in the dark for 2 h. The fluorescence staining was observed under laser scanning confocal microscope.

### 2.9. Immunohistochemical Staining [23]

The tissue slices of nude mice with LC were obtained, dried 1 h at 60°C, dewaxed with xylene, and rehydrated with ethanol fractionation. The antigen repair was processed with citrate buffer (pH 6.0), autoclaved and sterilized at 121°C, washed with PBS, and sealed with goat serum (Boster, Wuhan) at ambient temperature for 30 min. The slices were cultivated with IDO1 and CD8+ antibodies at 4°C overnight or TUNEL apoptosis assay colorimetric kit (Beyotime, Shanghai, China) at 37°C for 60 min. Then, it was washed by PBS and sliced. Polink-1 HRP DAB and one-step polymer detecting systems were used to incubate at ambient temperature for 20 min. Lastly, the slides were counterstained with hematoxylin. The positive staining cells were counted in five stochastically selected regions, and the average of positive staining cells in each region was calculated. Image-Pro Plus 6.0 was used to quantitatively analyze the staining of IDO1, CD8+, and TUNEL (apoptotic markers).

### 2.10. Isolation and Culture of White Blood Cells

Human white blood cells were obtained by separating peripheral blood. The test tubes of ethylenediaminetetraacetic acid were used for subpackaging and analysis. At room temperature, it was centrifuged at 500 × *g* for 10 min and the supernatant was discarded. The volume of ACK lysis buffer solution (10 times) was added. It was then lightly swirled for 5 min and centrifuged (500 × *g*, 10 min), and the supernatant was discarded. The procedure was repeated until all erythrocytes were completely removed. Finally, leukocytes were collected. Under the condition of RPMI 1640 with 10% FBS, the cells were regulated to 4 × 10^6^ cells/ml. The miR-760-mimics or the control group was transfected into A549 and H1299 cells at 30 ng/ml IFN-*γ*, respectively (GenScript, China). IFN-*γ* was treated for 24 h and used as conditioned medium (CM). Then, we collected the supernatant after cell culture. The leukocytes (100 *μ*l) were inoculated into the 96-well plate, and then, different CM (100 *μ*l) was put in the 96-hole plate and cultivated for 48 h.

### 2.11. Analysis of Flow Cytometry

The leukocytes cultured in different CM for 48 hours were collected, resuspended with PBS, and dyed 15 min with FITC anti-human CD8+ in the dark at 4°C. Cells were centrifuged and suspended in binding buffer. The annexin V-APC/7-AAD double dyeing was performed with annexin V-APC/7-AAD apoptosis kit, and the staining method was carried out based on the kit instructions. In addition, tumor tissues of mice were separated by using the Tumor Dissociation Kit and then adjusted to single cell suspension. The single cell suspension was stimulated with BD white blood cell activation mixture (No. 550583) for 5 h. The tumor cells were dyed for 0.5 h with the Zombie Yellow™ Fixable Viability Kit. Then, the cells were dyed with CD45, CD4, and CD8+ for 0.5 h. After immobilization and permeabilization, the cells were fluorescently dyed with Foxp3. Cytek Aurora flow cytometer and FlowJo were used. The apoptosis was tested via annexin V-FITC apoptotic kit (BD Biosciences, Erembodegem, Belgium). Cells were obtained, rinsed twice through cold PBS, and resuspended in annexin V binding buffer. After that, they were dyed 15 min through fluorescein isothiocyanate (FITC) and propidium iodide (PI) at 4°C.

### 2.12. Double Luciferase Report

The bioinformatics analysis tools were applied (TargetScan (http://www.targetscan.org/vert_72/) and miRDB (http://mirdb.org/)). The luciferase pmirGLO reporter vector was performed for constructing IDO1-wild type 3′-UTR (IDO1-wt) and IDO1 mutant 3′-UTR (IDO1-mut). Cells were inoculated into a 12-hole plate at 1 × 10^5^ per hole, cultivated for one night, and cotransfected with 100 nmol of miR-760-mimics or control group plus 100 ng of pmirGLO-30-UTR. The UTR plasmid of Lipofectamine 3000 (Invitrogen) was used for 48 h. The luciferase activity was tested via a dual-luciferase reporter (Promega Corporation, Madison, WI, the United States).

### 2.13. Statistical Analysis

The required pictures were drawn and data were assessed via GraphPad 8. The measuring data were marked as mean number ± standard deviation (mean ± SD) and compared through independent sample *t* test. The counting data were shown as percentage (%) and tested by chi-squared test, represented as *χ*^2^. One-way analysis of variance was employed for multigroup comparison, marked by F. LSD-t test was applied for pairwise comparison afterward. Multiple time points were analyzed by repeated measures analysis of variance and marked by F. Bonferroni was used for back testing. The correlation of miR with mRNA in patients' tumor tissues was analyzed. The relationship of miR-760 with survival was analyzed by K-M test (*P* < 0.05).

## 3. Results

### 3.1. miR-760 Was Reduced in NSCLC Patients with Unfavourable Prognosis

The miR-760 in NSCLC patients was first tested by qRT-PCR. The results manifested that the miR-760 in the tumor tissues of NSCLC patients was downregulated compared with the adjacent tissues (Figure 1(a). Further analysis denoted that reduced miR-760 level was bound up with the tumor stage of NSCLC (Figure 1(b). Furthermore, patients were separated into high and low expression groups on the basis of miR-760's median value [24, 25]. miR-760 was discovered to be unrelated to age, gender, tumor size, or differentiation, although it was related to TNM stage and lymphatic metastasis (Table 1). In addition, we followed up with the patients. By January 2019, all patients had been followed up on, and no follow-ups had been missed. It was observed that the total survival time of low-expressed miR-760 patients was obviously lower than that of those with high expression (Figure 1(c). Therefore, miR-760 was a latent prognostic index for NSCLC patients. qRT-PCR detection manifested that the miR-760 in LC cell strains also showed a downward trend (Figure 1(d). This indicated that miR-760 might affect the development and progress of LC.

### 3.2. miR-760 Affects LC Development and Progression

To ascertain miR-760's mechanism in LC, we carried out cell experiments in vitro. At first, we established miR-760-mimics and miR-760-inhibit vectors, respectively, and transfected them into A549 and H1299 cells. It turned out that the miR-760 enhanced after transfection of miR-760-mimics, but it reduced obviously after transfection of miR-760-inhibit (Figure 2(a). Then, we tested the growth, invasiveness, migration, and apoptosis of cells transfected with miR-760-mimics and miR-760-inhibit by CCK-8, Transwell, and FACS, respectively. CCK-8 test revealed that the proliferation of cells transfected with miR-760-mimics was obviously inhibited compared with the control group, while the growth of cells with miR-760-inhibit was obviously enhanced (Figure 2(b). Transwell experiment also denoted that cell invasion and migration after transfection of miR-760-mics reduced obviously compared with the control group, while those after transfection of miR-760-inhibit enhanced obviously (Figures 2(c) and 2(d). In addition, FACS experiments also showed that apoptosis was induced after transfection with miR-760-mimics, while the apoptosis rate reduced after transfection with miR-760-mimics (Figure 2(e). These experiments confirmed that miR-760 affected the occurrence of LC and it was a latent therapeutic target in clinic.

### 3.3. There Was a Targeted Relationship of miR-760 with IDO1

miR regulated downstream target genes to take part in tumor development. We concluded that there was a targeted connection of IDO1 with miR-760 through online prediction analysis. At first, we tested the IDO1 mRNA and protein in LC cell strains after transfection of miR-760-mimics and miR-760-inhibit by qRT-PCR and WB. It manifested a significant regulatory effect (Figures 3(a) and 3(b). Then, we further detected the IDO1 in tumor tissues of NSCLC patients. The findings signified that the IDO1 in tumor tissues of NSCLC patients increased obviously (Figure 3(c). Correlation analysis concluded that miR-760 was positively correlated with the IDO1 relative expression in tumor tissues of NSCLC patients (Figure 3(d). There was a targeted regulatory relationship of miR-760 with IDO1. Then, the double luciferase reporter revealed that miR-760-mimics suppressed IDO1-wt fluorescence activity, while miR-760-inhibit upregulated the fluorescence activity of IDO1 (Figures 3(e)–3(g). It could be concluded that miR-760 and IDO1 were targetly related.

### 3.4. Upregulating miR-760 Could Reverse LC Cell Growth and Metastasis Induced by Overexpression of IDO1

miR-760 was tested in rescue experiments to see if it had a role in LC cell growth and progression through regulating IDO1. The following were our initial findings. A549 and H1299 cells were transfected with pcDNA-IDO1, which promoted LC cell proliferation, invasiveness, and migration while suppressing apoptosis. However, the above effects were reversed after miR-760-mimics and pcDNA-IDO1 cotransfection; that is, cell growth, invasiveness, and migration were obviously accelerated, and apoptosis was promoted. So, miR-760 could regulate IDO1 to take part in LC development (Figure 4).

### 3.5. IFN-*γ* Improved the Survival of CD8+ T Cells by Inhibiting miR-760 and Upregulating IDO1

Early studies have shown that IFN-*γ* can upregulate IDO1 in LC cells. Moreover, IDO1 also affects tumor immunity. Tumor occurrence and development are influenced by the tumor immunological microenvironment. Treg cells, a type of lymphocyte subgroup with immune regulation function, keep the immune system in check and prevent illnesses, particularly by boosting tumor progression and helping tumor escape. Therefore, we have speculated that miR-760/IDO1 axis may also play an immunomodulatory role in LC. First, we analyzed the effect of miR-760 upregulation on the CD8+ T level and found that the number of CD8+ T cells in the miR-760-mimic group increased. Then, we transfected miR-760-mimics or control group into A549 and H1299 cells at 30 ng/ml IFN-*γ*. By detecting the apoptosis ratio of CD8+ T cells, FACS revealed that compared with NC group without IFN-*γ* treatment, the percentage of apoptotic CD8+ T cells treated with control group and IFN-*γ* increased. However, compared with the NC group, the percentage of apoptotic CD8+ T cells in miR-760-mimics group was relatively lower, which indicated that miR-760 heightened the survival rate of CD8+ T cells (Figures 5(a) and 5(b)), suggesting that miR-760 could mediate IDO1 to regulate CD8+ T cell apoptosis.

### 3.6. miR-760 Mediated IDO1 to Inhibit CD8+ T Cell Reaction in Tumor Tissues of Nude Mouse

To further evaluate the regulatory effect of the miR-760/IDO1 axis on CD8+ T apoptosis, we created an in vivo model. To observe tumor formation, nude mice were injected subcutaneously with lentivirus transfected and stably expressed pLV-THM-miR-760 or pLV-THM-miR-NC A549 cells. The findings manifested that the tumor volume of nude mice in pLV-THM-miR-760 group gradually decreased compared with pLV-THM-miR-NC group with the increase of time. The nude mice were killed and the quality of tumor tissue was compared after 28 days. It was also found that the quality of tumor tissue in pLV-THM-miR-760 group was obviously lower than that in pLV-THM-miR-NC group. What is more, qRT-PCR and WB denoted that the miR-760 level of nude mice tissue increased in pLV-THM-miR-760 group, while the IDO1 mRNA and protein level decreased. Furthermore, we further explored through IHC technology and found that after pLV-THM-miR-760 intervention, the number of IDO1+ cells was lower than that in pLV-THM-miR-NC group, and that of CD8+ T cells in tumor tissues after pLV-THM-miR-760 intervention was obviously higher than that in the pLV-THM-miR-NC group. Immunofluorescence staining found that IDO1 was localized in cytoplasm, mainly in tumors. CD8+ was localized on lymphocyte membrane, and CD8+ in cells was observed. The results of IDO1 staining were consistent with IHC. At this point, we proved that miR-760 could promote CD8+ T cell apoptosis by downregulating IDO1, thus inhibiting the immune escape of cells (Figure 6).

## 4. Discussion

LC is one of the main reasons of carcinoma death, and there is no good treatment plan at present [26, 27]. In our research, we experimentally confirmed that miR-760 was low expressed in LC and it promoted CD8+ cell apoptosis by regulating IDO1. It provides a potential theoretical foundation for the development of new immunization therapy in treating LC.

miR is a short-chain noncoding RNA. Research has manifested that miR is relevant to LC development and progression [28]. miR-760 is a familiar tumor suppressor gene with low expression in esophageal cancer [29], ovarian cancer [30], and liver cancer [31]. miR-760's mechanism in LC was not reported. Therefore, this research was devised to analyze the related mechanisms of miR-760 in LC. We first analyzed the miR-760 in tumor tissues of NSCLC patients. And we concluded that the miR-760 in tumor tissues of NSCLC patients and LC cell strains decreased obviously. Further analysis revealed that the miR-760 reduced gradually with the increase of TNM stage, which uncovered that miR-760 might be related to the occurrence of LC. Besides, we analyzed the connection of miR-760 with clinical data and discovered that the incidence of high TNM stage and lymphatic metastasis increased in low-expressed miR-760 patients. K-M survival analysis revealed that the overall survival rate of patients with low expression of miR-760 reduced. These studies proved that miR-760 was a latent prognostic index of NSCLC.

In clinic, encouraging apoptosis and slowing tumor development are significant techniques for treating tumors [31]. The LC cell lines transfected with miR-760-mimics and miR-760-inhibit were created to evaluate miR-760's influence on LC cell development and progression. We discovered that upregulation of miR-760 inhibited cell growth, invasion, and migration, as well as induced apoptosis, in experiments. However, when miR-760 was inhibited, the above results were reversed, indicating that miR-760 was involved in cell development and progression and could be a therapeutic target. To better seek the potential mechanisms of miR-760, we conducted online prediction site analysis and discovered that there might be a targeting relationship between IDO1 and miR-760. IDO1 is an immunomodulatory enzyme, which can induce apoptosis/dysfunction of effector T cells and produce immunosuppressive regulatory T cells [32]. To verify their regulatory relationship, we tested the IDO mRNA and protein relative expressions in cells transfected with miR-760-mimics and miR-760-inhibit via qRT-PCR and WB experiments, respectively. The findings showed that the IDO mRNA and protein in cells was regulated after overexpression or inhibition of miR-760. We speculated that there might be a targeting relationship between IDO1 and miR-760. Then, we verified our hypothesis by double luciferase report. In addition, we also confirmed that IDO1 was highly expressed in tumor tissues of NSCLC patients and negatively correlated with miR-760, which also verified our results from the side. Furthermore, the cell experiments denoted that cell growth, invasiveness, and migration were enhanced after transfection of pcDNA-IDO1, and the decrease of apoptosis rate was saved after miR-760-mimics cotransfection. All these experiments indicated that miR-760 participated in the development of LC by regulating IDO1.

Research has shown that the functional inactivation of tumor-reactive T cells may be an important mechanism to escape tumor immunity [33]. Early studies have shown that [34] IDO1 can promote tumor immune escape. IFN-*γ* is a crucial cytokine produced by activated T cells, natural killer cells (NK), and NK T cells in tumor microenvironment, and it exerts vital effects in coordination process [35, 36]. In addition, early studies have shown that [37, 38] IFN-*γ* can activate IDO1, which can promote CD8+ cell apoptosis and realize immune escape. In order to explore whether miR-760 can regulate IDO1 to participate in tumor immune response, 30 ng/ml of IFN-*γ* was cocultured with LC cells transfected with miR-760-mimics. It manifested that the apoptosis rate of CD8+ cells in LC increased obviously in the IFN-*γ*+mimics-NC group, but the apoptosis of CD8+ cells was inhibited after coculture, suggesting that upregulating miR-760 suppressed CD8+ cell apoptosis by inhibiting IDO1, thus inhibiting tumor immune escape.

To further understand the mechanism of miR-760 in LC, we created an in vivo model. It was discovered that miR-760 grew significantly in tumors of naked mice, indicating that the in vivo model had been successfully developed. Further detection of tumor volume and mass in nude mice manifested that the tumor volume and mass were significantly inhibited in pLV-THM-miR-760 group compared with the control group. Furthermore, the IDO1 mRNA and protein relative in tumor tissues was also significantly inhibited.

Nevertheless, there are still some shortcomings in this research. First of all, IDO1 can induce apoptosis/dysfunction of T cells by catalyzing tryptophan degradation to kynurenine. Unfortunately, these two indicators were not detected in this study. Secondly, we did not test the IDO1 protein in tumor tissues of NSCLC patients in this research. Early researches have revealed that IDO1 protein is highly expressed in colon cancer, but there is no difference in IDO1 mRNA level between colon cancer and normal tissues. For this reason, we will conduct more basic experiments to continuously enrich our conclusions.

## 5. Conclusion

Evidence showed that IDO-1 not only participates in the immune escape process of lung cancer but also contributes to the safety of the pretumor area. In addition, studies have shown that IDO-1 can induce immunosuppression and promote tumor progression in LC animal models. Overall, upregulating miR-760 can inhibit the apoptosis-promoting effect of IDO1 on CD8+, thus inhibiting tumor immune escape, which is a latent strategy for treatment and new drug development.

## Figures and Tables

**Figure 1:** miR-760 level and prognosis in NSCLC patients. (a) The miR-760 level in NSCLC patients is tested via qRT-PCR. (b) The miR-760 level in different stages of NSCLC patients is tested via qRT-PCR. (c) The total survival of patients in miR-760 high and low expression groups is assessed via K-M survival. (d) The miR-760 level in LC cell lines is tested via qRT-PCR. ^∗^*P* < 0.05, ^∗∗^*P* < 0.01, and ^∗∗∗^*P* < 0.001.

**Figure 2:** miR-760's effect on LC cell growth and development. (a) The miR-760 level in LC cells after transfection of miR-760-mimics and miR-760-inhibit is tested via qRT-PCR. (b) LC cell proliferation after transfection of miR-760-mimics and miR-760-inhibit is tested via CCK-8. (c and d) The number of LC cells invasion and migration after transfection of miR-760-mimics and miR-760-inhibit is assessed via Transwell test. (e) The apoptosis rate of LC cells after transfection of miR-760-mimics and miR-760-inhibit is assessed via FACS test. ^∗^*P* < 0.05 and ^∗∗^*P* < 0.01.

**Figure 3:** miR-760 could target IDO1. (a) The IDO1 mRNA level in cells transfected with miR-760-mimics/miR-760-inhibit is tested via qRT-PCR. (b) The IDO1 protein level in cells transfected with miR-760-mimics/miR-760-inhibit is tested via WB. (c) The IDO1 level in tumor tissues of NSCLC patients is tested via qRT-PCR. (d) The correlation between IDO1 and miR-760 in tumor tissues of NSCLC patients is assessed via Pearson test. (e) Binding and mutation sites of miR-760 and IDO1. (f and g) Dual-luciferase reporter confirmed that miR-760 had target correlation with IDO1. ^∗^*P* < 0.05 and ^∗∗∗^*P* < 0.001.

**Figure 4:** miR-760 targeted IDO1 to inhibit LC cell growth. (a) Cell proliferation after cotransfection of miR-760-mimics and pcDNA-IDO1 is tested via CCK-8 experiment. (b and c) Cell invasion and migration after cotransfection of miR-760-mimics and pcDNA-IDO1 are assessed via Transwell test. (d) The apoptosis rate after cotransfection of miR-760-mimics and pcDNA-IDO1 is tested via FACS. ^∗^*P* < 0.05.

**Figure 5:** IFN-*γ* improved CD8+ T cell survival by regulating miR-760/IDO1 axis. (a) CD8+ T cell survival after A549 cell coculture. (b) CD8+ T cell survival after H1299 cell coculture. ^∗^*P* < 0.05 and ^∗∗^*P* < 0.01.

**Figure 6:** Upregulating miR-760 inhibited CD8+ T cells in tumor through IDO1. (a) Changes of tumor volume within 28 days of the tumorigenesis experiment. (b) Comparison of tumor mass in nude mice killed at 28 days. (c) The miR-760 and IDO1 levels in tumor tissues of nude mice are tested via qRT-PCR. (d) The IDO1 protein level in tumor tissues of nude mice is tested via WB. (e) Immunohistochemical staining of IDO1 and CD8+ in tumor tissue sections of nude mice in pLV-THM-miR-760 or pLV-THM-miR-NC group. ^∗^*P* < 0.05 and ^∗∗∗^*P* < 0.001.

**Table 1:** Relationship between miR-760 and clinical data of patients.

Factors		miR-760 relative level		*P* value
		Low expression (*n* = 26)	High expression (*n* = 26)	
Gender				0.578
	Male (*n* = 28)	13	15	
	Female (*n* = 24)	13	11	

Age				0.397
	≥60 years old (*n* = 21)	9	12	
	<60 years old (*n* = 31)	17	14	

Tumor size				0.405
	≥5 cm (*n* = 27)	12	15	
	<5 cm (*n* = 25)	14	11	

Differentiation				0.560
	Poorly differentiated (*n* = 18)	10	8	
	Middle+well differentiated (*n* = 34)	16	18	

Lymphatic metastasis				0.032^∗^
	Metastasis (*n* = 15)	11	4	
	Nonmetastasis (*n* = 37)	15	22	

TNM staging				0.039^∗^
	I+II (*n* = 35)	14	21	
	III+IV (*n* = 17)	12	5	

Note: ∗ means *P* < 0.05, and there were differences between groups.

## Data Availability

The datasets used and/or analyzed during the current study are available from the corresponding author on reasonable request.
